# *Astragalus membranaceus* and *Salvia miltiorrhiza* Ameliorate Hypertensive Renal Damage through lncRNA-mRNA Coexpression Network

**DOI:** 10.1155/2022/3002353

**Published:** 2022-09-09

**Authors:** Le Zhou, Cong Han, Yao Liu, Tao Cui, Zhen Shen, Xiang-yu Li, Yue-hua Jiang, Wei Li

**Affiliations:** ^1^Shandong University of Traditional Chinese Medicine, Jinan 250014, China; ^2^Department of Nephropathy, Affiliated Hospital of Shandong University of Traditional Chinese Medicine, Jinan 250014, China; ^3^Central Laboratory of Affiliated Hospital of Shandong University of Traditional Chinese Medicine, Jinan 250014, China

## Abstract

lncRNAs and mRNA are closely associated with hypertensive renal damage, and *Astragalus membranaceus* and *Salvia miltiorrhiza* (AS) have a therapeutic effect; however, the mechanism of AS to ameliorate hypertensive renal damage through the co-expression network of lncRNA-mRNA was unclear. In this study, we investigated the role of AS regulated the coexpression network of lncRNA-mRNA in improving hypertensive renal damage. Sixteen 24-week old spontaneous hypertensive rats (SHRs) were randomly divided into model group (*M*) and drug intervention group (AS, 5.9 g/kg), 8 Wistar Kyoto rats (WKY) of the same age as normal group (*N*). The treatment of rats was 4 weeks. Detecting the change of blood pressure, renal pathology and renal function related indicators, and lncRNA and mRNA sequencing and joint analysis was performed on the kidney. AS reduced blood pressure; decreased urine NAG, urine mALB, serum CysC, and IL-6; and improved renal pathology compared with group M. Simultaneously, AS reversed the disordered expression of 178 differential expression (DE) mRNAs and 237 DE-lncRNAs in SHRs, and their joint analysis showed that 13 DE-mRNAs and 32 DE-lncRNAs were coexpressed. Further analysis of 13 coexpressed DE-mRNAs showed negative regulation of blood pressure and fatty acid beta-oxidation was highly enriched in GO pathways, *PPAR* signaling pathway was highly enriched in KEGG pathways, and the verification related to these pathways was also highly consistent with the sequence. AS can alleviate hypertensive renal damage through the coexpression network of lncRNA-mRNA, of which coexpressed 13 DE-mRNAs and 32 DE-lncRNAs were the important targets, and the pathway negative regulation of blood pressure, fatty acid beta-oxidation, and PPAR signaling pathway play a major regulatory role.

## 1. Introduction

Hypertensive renal damage, reversible in early stage, is related to hemodynamic changes, inflammation and oxidative stress, excessive renin angiotensin activation, genetic factors, and metabolic factors. Numbers of patients with end stage renal disease (ERSD) due to hypertension are increasing year by year, accounting for about 28% of all ESRD cases [1]. In-depth exploration of the pathogenesis of hypertensive renal damage and intervention measures is of great significance for delaying progress. lncRNA is a noncoding RNA that can directly or indirectly regulate mRNA expression by interacting with mRNA, thereby affecting post transcriptional genes and proteins [2]. lncRNAs are closely associated with hypertension and renal damage. For example, lncRNAs can participate in vascular remodeling by affecting endothelial cell proliferation and phenotypic transformation of vascular smooth muscle [3–6]. lncRNA-p21 enhances autophagy by promoting the transcriptional activity of p53 to prevent endothelial progenitor cells damage caused by AngII [7]. High expression of H19 could downregulate the expression of fibronectin and destroy the integrity of renal vessels [8], and lncRNA MALAT1 promoted transforming growth factor-*β*1 (TGF-*β*1), induced endothelial to mesenchymal transition (EndMT) of endothelial progenitor cells (EPCs), and accelerated renal fibrosis [9, 10]. However, the role of the coexpression network of lncRNAs and mRNAs in hypertensive renal damage has not yet been fully clarified.

In traditional Chinese medicine (TCM), *Astragalus membranaceus* (AM, of the Leguminosa family) has the function of Tonifying Qi. *Salvia miltiorrhiza* (SM, of the Lamiaceae family) could promote blood circulation and remove blood stasis. Previous studies have shown that both AM and SM could relax blood vessels and resist oxidative stress and anti-inflammatory [11–13]. *Astragalus membranaceus* and *Salvia miltiorrhiza* (AS) are often used to treat hypertensive renal damage as a representative of invigorating qi and promoting blood circulation in TCM. We have found that AS can not only reduce blood pressure through intestinal flora-host metabolism [14] but also improve hypertensive renal damage by regulating phosphoinositide 3-kinases (PI3K)/serine-threonine protein kinase 1 (AKT1) and TGF-*β*1 pathways [15, 16]. However, the mechanism of AS to ameliorate hypertensive renal damage through the coexpression network of lncRNA and mRNA was unclear.

In this study, we mainly investigated the mRNAs and lncRNAs in the kidney of SHRs and the effect of AS on the coexpression profile, so as to clarify the main target and related pathways of AS in the treatment of hypertensive renal damage.

## 2. Materials and Methods

### 2.1. Extraction and Identification of AS

AM and SM (AS) were provided by the Affiliated Hospital of Shandong University of TCM. The preparation and quality control of AS were based on our previous research [14, 17]. Briefly, AM and SM were mixed in a ratio of 2 : 1, 10 times the volume of water was added to soak for 1 hour and then decocted for 30 minutes. After filtration and extraction of filtrate, filtrate was extracted from filtrate residue again according to the same procedure, and the two filtrate were mixed to obtain AS solution of 0.59 g crude drug per ml [14]. Finally, the main components of AS were identified and analyzed by UPLC- MS/MS [17].

### 2.2. Preparation of Animals

Animals were purchased from Vital River Laboratory Animal Technologies Co., Ltd. (no. SCXK (Beijing) 2016-0006). The project has passed the review of ethics committee of Affiliated Hospital of Shandong University of TCM. 16 male SHRS aged 24 weeks were divided into model group (*M*, *n* = 8) and drug intervention group (AS, *n* = 8) as random, and the control group (*N*) consisted of 8 age-matched WKY rats. The AS group was given AS (5.9 g/kg, referring to the dose of AS commonly used in clinical patients [14]) by intragastric administration, and the *M* and *N* groups were given equal volume of normal saline. The rats were intragastric once daily for 4 weeks.

### 2.3. Blood Pressure Measurement and Sample Collection

We used a noninvasive sphygmomanometer (ALC-NIBP System, Alcott BioScientific) to measure the blood pressure (BP) of rat caudal artery before and 1, 2, 3, and 4 weeks after intervention. The rats were anesthetized, serum was collected after 4 weeks of intervention, and the serum was centrifuged at a speed of 3000 r/min for 10 minutes and then stored at low temperature (-80°C). Rat kidney tissue was obtained and fixed with formaldehyde for 48 hours. After paraffin embedded, sections in 4 *μ*m thick were cut.

### 2.4. Biochemical Analysis and Pathological Staining

Automatic biochemical analyzer (Rayto, China, Chemray240) was used to determine serum creatinine (Scr) and blood urea nitrogen (BUN) levels. Urine microalbumin (mALB), urine N-acetyl-*β*-D-glucosidase (NAG), serum cystatin C (CysC), and interleukin-6 (IL-6) were determined by enzyme-linked immunosorbent assay (ELISA), haematoxylin-eosin (HE) staining, and Masson trichrome staining process paraffin sections, which were observed under light microscopic.

### 2.5. Transcriptome Sequencing and Analysis

#### 2.5.1. Library Construction and Sequencing

The RNeasy mini kits were used to isolate the RNA, and strand-specific libraries were prepared using the VAHTS Total RNA-seq (H/M/R) Library Prep Kit (Vazyme, China). In Brief, RNA was purified after removal of rRNA by magnetic beads. The cleaved RNA fragments, which were segmented with divalent cations(94°C, 8 min), were used to synthesize the first strand cDNA; then, the reverse transcriptase and random primers were used to generate the second strand cDNA. After PCR purification and enrichment, the final cDNA library was generated. Then, Qubit® 2.0 Fluorometer (Life Technologies, USA) was used for quantification, and Agilent 2100 biological (Agilent Technologies, USA) was used for verification, so as to determine the size of the insert and calculate the molar concentration. cBot was used for cluster analysis, and Illumina NovaSeq 6000 (Illumina, USA) was sequenced. Shanghai Sinomics Corporation constructed and sequenced the library.

#### 2.5.2. Analysis of lncRNA and mRNA

The offline reading of sequencing was preprocessed. Alignment was performed with Hisat2 software, so clean reads could mapped to the Rnor6.0.91 reference genome. StringTie was then run with a reference annotation to generate FPKM values differentially expressed (DE) lncRNAs and DE-mRNAs. The *P* value significance thresh for known gene models. Display differences based on fold change (FC) and false discovery rate (FDR). DE-mRNAs and DE-lncRNAs were set to FC > 1.5 or <0.67 and *P* < 0.05, and further combined analysis was shown in the network diagram. Specifically, genes transcribed within 10-kbp window upstream or downstream of the pancreas were considered to be cis-acting targets, and trans-acting target genes were identified by RNAplex software. Gene Ontology (GO) and Kyoto Encyclopaedia of Genes and Genomes (KEGG) pathway analysis were used to analyze the functions of the coexpressed DE-mRNAs.

### 2.6. Quantitative Real-Time Polymerase Chain Reaction (qRT-PCR) Analysis of lncRNAs and mRNAs

We used the FastPure total RNA isolation kit (Vazyme, Nanjing, China, RC101) to extract total RNA. PrimeScriptTM RT kits were used to reverse-transcribed, and TB GreenTM Ex TaqTM kits were used to execute the qRT-PCR. RT-PCR was performed using a Light Cycler480 II instrument (Roche, Germany). lncRNAs and mRNAs were normalized using the expression of GAPDH, and the relative RNA levels were analyzed by2-*ΔΔ*CT method. Gene-specific primer sequences of genes (Sparkjade, China) were designed and listed that in Table 1.

### 2.7. Statistical Analysis

Statistical analyses were performed with SPSS 21.0. The data were described as the mean ± standard deviation (SD). Differences between groups were analyzed by one-way ANOVA, and differences were considered significant if *P* values less than 0.05.

## 3. Results

### 3.1. AS Ameliorated Blood Pressure and Renal Function

After 3 weeks, the diastolic blood pressure (DBP) of AS group was significantly lower than the M group (*P* < 0.05). Systolic blood pressure (SBP) and DBP in AS group were both lower than M group (*P* < 0.05) 4 weeks later (Figure 1(a)). In addition, compared to group *N*, urine NAG which is reflected to renal tubular injury and urine mALB in response to proteinuria was both increased in *M* group (*P* < 0.01), and both were improved by AS (*P* < 0.05 or *P* < 0.01) (Figures 1(b) and 1(c)). There was no significant change in Scr and BUN among three groups, serum CysC increased in group M, which reflects early renal function injury and was recalled by AS (*P* < 0.05) (Figures 1(d) and 1(f)). Besides, AS decreased IL-6 compared with group *M*, which represented the inflammatory level (*P* < 0.05 or *P* < 0.01) (Figure 1(g)).

### 3.2. The Effect of AS on Renal Pathology

The renal pathology that may lead to the deterioration of renal function was further explored. HE staining of rats in the M group showed hyaline degeneration of small arteries, dilation of renal tubules, vacuolation of cytoplasm, and tubule atrophy. Masson staining showed that the renal interstitium was widened and fibrotic. TUNEL showed that apoptosis was increased. AS improved the above pathological injury in varying degrees (Figures 2(a)–2(c)).

### 3.3. AS Modified the Disordered lncRNA Expression Profiles

In the 3 groups, we performed lncRNA sequencing aiming to explore the role of SHRs in renal damages and the intervention targets of AS. Using the Volcano plots to show the lncRNA expression profiles after compared the group *M* to the other 2 groups. Among 1435 DE-lncRNAs (*M* vs. *N*), 700 were upregulated and 735 were downregulated (Figure 3(a)). Among 726 DE-lncRNAs (AS vs. *M*), 355 were upregulated and 371 downregulated (Figure 3(b)). 237 DE-lncRNAs were found to be shared and showed the same trend in two comparisons with group *M* after further cluster analysis (Figure 3(c)), suggesting that they are important targets for SHR as to reverse renal injury lncRNAs.

### 3.4. AS Regulated the Coexpression Network and Pathways of lncRNA-mRNA

SHRs regulated the genetic by further transcriptome sequencing in the same kidney. In group *N*, 1786 DE-mRNAs were found, 1097 were upregulated and 689 downregulated compared to group *M* (Figure 4(a)). In group AS, 596 DE-mRNAs were found, 246 were upregulated and 350 downregulated (Figure 4(b)). 178 DE-mRNAs had a common change trend in the comparison between the other two groups and group *M*, which were displayed by cluster analysis (Figure 4(c)). Furthermore, we performed an association analysis between 237 DE-lncRNAs and 178 DE-mRNAs and constructed a coexpression network of the two. Then, 13 DE-mRNAs were predicted by 32 DE-lncRNAs, and their coexpression network map was further constructed (Figure 5). Finally, we performed KEGG and GO enrichment analysis on 13 DE-mRNAs. Three pathways positive regulation of blood pressure, negative regulation of blood pressure, and fatty acid beta-oxidation were highly enriched in GO analysis. In addition, pathway PPAR signaling pathway was highly enriched in KEGG analysis (Figure 6). Specific information of coexpressed 13 DE-mRNAs and 32 DE-lncRNAs among the three groups is listed in Table 2.

### 3.5. Validation of Coexpression of DE-lncRNAs and DE-mRNAs Regulated by AS

8 coexpressed DE-lncRNAs were further verified. The expression of NONRATT028523.2, NONRATT028522.2, MSTRG.22291.30, NONRATT022172.2, and ENSRNOT00000083625 increased in *M* group and decreased in varying degrees after AS intervention. At the same time, the expression of NONRATT026955.2, NONRATT016111.2 and MSTRG.15507.1 in *M* group decreased, which was also recalled by AS (Figures 7(a)–7(h)). We further verified 7 coexpressed DE-mRNAs. The expression of Adipoq and Abcd2 decreased, and the expression of Lpl, Cnr1, Fst, Mapk13, and Zbtb16 increased in *M* group, which were reversed by AS (Figures 8(a)–8(g)). All the verification were consistent with the sequencing results.

## 4. Discussion

Our study showed that AS could not only lower blood pressure steadily but also improve the damage of renal structure and function in SHRs. Specifically, on the one hand, AS reduced the levels of urine NAG, urine mALB, serum CysC, and IL-6 and increased the level of SOD, which indicated that AS can effectively abate proteinuria, relieve the damage of early renal function, and regulate the level of inflammation and oxidative stress as a whole. On the other hand, AS improved glomerular basement membrane thickening, renal tubular dilatation, and vacuolar degeneration in SHRs, which was consistent to our previous study [15, 16]. Furthermore, we found for the first time that AS inhibits collagen fibroplasia and apoptosis in renal tissue to some extent. Then, we further searched for the mechanism of AS to lower blood pressure and improve renal damage from the coexpression network of mRNAs and lncRNAs. AS reversed the disordered expression of 237 DE-lncRNAs and 178 DE-mRNAs in SHRs found in sequencing. lncRNAs can directly regulate mRNA and participate in the process of hypertension or kidney damage. Therefore, we conducted an association analysis on 237 DE-lncRNAs and 178 DE-mRNAs, and the results showed that 13 DE-mRNAs and 32 DE-lncRNAs were coexpressed, which were important targets of AS. Further analysis of 13 coexpressed DE-mRNAs indicated that PPAR signaling pathway was highly enriched in KEGG pathways, and negative regulation of blood pressure and fatty acid beta-oxidation was highly enriched in GO pathways.

Our previous studies *in vitro* found that PPAR signaling pathway and renin-angiotensin system were highly involved in Ang II induced injury of renal arterial endothelial cells (RRAECs) by integrative analysis of miRNA-mRNA sequencing [18]. This study *in vivo* found that PPAR signaling pathway was also closely involved in the regulation of AS on BP and renal damage in SHRs. PPARs have key regulatory roles in metabolism, hypertension, and vascular function and comprise three subtypes, PPAR *α*, *γ*, and *β*/*δ*. PPAR *γ* could inhibit the oxidative stress of vascular endothelial cells and antagonize the renin-angiotensin system of vascular smooth muscle cells to relax blood vessels during hypertension [19]. In hypertensive nephropathy, gastrin normalized blood pressure, reduced renal tubular cell apoptosis, and increased macrophage endocytosis by activating PPAR *α* [20], and PPAR*β*/*δ*-dependent vasodilator pathway can selectively control renal blood flow [21]. Our sequencing results showed that Adipoq and lipoprotein lipase(Lpl), the important downstream effectors of PPAR *α*, *γ* and *β*/*δ*, were decreased in SHRs and were recalled by AS. Adipoq, which was the target gene of 8 DE-lncRNAs such as MSTRG.15507.1 and MSTRG.22291.30, played a role of renal protective agent by inhibiting renal inflammation, oxidative stress, reducing albuminuria and kidney fibrosis as an endogenous bioactive polypeptide or protein secreted by adipocytes in DCA + Ang II-induced CKD mice [22, 23]. Serum Adipoq levels in patients with pregnancy-induced hypertension were negatively correlated with albuminuria [24]. In addition, Lpl, the target gene of ENSRNOT00000083625, not only aggravated the early development of type 1 diabetic nephropathy in mice but also resulted in lipid accumulation in nephrotic syndrome and CKD [25, 26]. We verified by PCR that AS increased the expression of Adipoq and MSTRG.15507.1 and decreased the expression of Lpl, MSTRG.22291.30, and ENSRNOT00000083625. This was highly consistent with the sequencing results and may be important targets for AS to improve hypertensive renal damage through PPAR signaling pathway.

Positive regulation of blood pressure, negative regulation of blood pressure, and fatty acid beta-oxidation were the top 3 pathway in go enrichment. Sequencing results showed that Cannabis receptor 1 (Cnr1), the target gene of NONRATT022172.2, which belongs to positive regulation of blood pressure, negative regulation of blood pressure pathway, increased in SHRs. Related studies have found that Cnr1 was expressed in many cell types of normal kidneys. Inhibiting its expression can not only regulate blood pressure by maintaining water and sodium balance but also delay the fibrosis of metabolic and nonmetabolic nephropathy [27]. Consistent with the results of sequence, AS reduced the expression of Cnr1 and NONRATT022172.2 by PCR, and the regulation of these two may be an effective mechanism for reducing the blood pressure of SHRs and protecting the kidneys. Fatty acid oxidation, especially *β*-oxidation of fatty acids in peroxisomes and mitochondria, was the main energy source for renal tubular epithelial cells. In CKD, the lack of key genes such as acyl-Coenzyme A oxidase (Acox) and phosphoenolpyruvate carboxy kinase (PCK) for fatty acid *β*-oxidation can directly induce ATP depletion, apoptosis, and lipid accumulation ultimately lead to epithelial-mesenchymal transition (EMT) and renal fibrosis [28, 29]. Sequencing results revealed that ATP binding cassette subfamily D member 2 (Abcd2), which was the target gene of 5 DE-lncRNAs such as NONRATT026955.2 and involved in peroxisomal import of fatty acids and/or fatty acyl-CoAs in the organelle [30], had a decreased expression in SHRs and was recalled by AS. Consistent with the sequence, AS increased Abcd2 and NONRATT026955.2 in the PCR verification, which may also contribute to the inhibition of renal tissue apoptosis by AS.

In addition, sequencing results also found that the expression of Fst, Prom2, RGD1561730, Syt13, Mapk13, Zbtb16, Usp9y, Slc4a7, and Nek5 in SHRs was disordered and recalled by AS. These genes were found to be related to the improvement of hypertensive renal damage by AS for the first time. The target gene Fst of NONRATT016111.2 belongs to the TGF-*β* signaling pathway, associated with renal fibrosis [31]. Zbtb16 is the target gene of NONRATT028523.2 and NONRATT028522.2 in the positive regulation of NK T cell differentiation pathway, whose overexpression can promote white fat production and accelerate lipid accumulation [32]. Our verification was highly consistent with sequencing and found that AS decreased the expression of Fst, Zbtb16, NONRATT016111.2, NONRATT028523.2, and NONRATT028522.2. In particular, the coexpression network confirms the molecular communication between genes. For example, Adipoq, Abcd2, and Mapk13 are regulated by MSTRG.15507.1 and MSTRG.22291.30 at the same time. Abcd2 and Mapk13 are also target genes of NONRATT026955.2. The mutual communication of coexpression differences may contribute to the improvement of hypertensive renal damage by AS.

In conclusion, the results of this study demonstrated that AS had good antihypertensive and renal protective effects, which may be mediated by the coexpression network of lncRNA-mRNA. This study provided new insights for *Astragalus membranaceus* and *Salvia miltiorrhiza* to improve hypertensive renal damage.

## Figures and Tables

**Figure 1:** Effects of AS on renal blood pressure and renal function. (a) Systolic blood pressure (SBP) and diastolic blood pressure (DBP). (b) Urine microalbumin (mALB). (c–f) Renal function related indicators: NAG: urine N-acetyl-*β*-D-glucosidase; BUN: blood urea nitrogen; Scr: serum creatinine; CysC: serum cystatin C. (g) Interleukin-6 (IL-6). Values are the mean ± SD (*n* = 8). ^#^*P* < 0.05, ^##^*P* < 0.01 vs. the *N* group. ^∗^*P* < 0.05, ^∗∗^*P* < 0.01 vs. the *M* group.

**Figure 2:** The effect of AS on kidney pathology (scale bars: 50 *μ*m, 400×). (a) HE staining (arrows points to lesions). (b) Masson staining (arrows represents collagen fibres). (c) TUNEL (green represents apoptotic cells).

**Figure 3:** Volcano plots and heat maps of DE-lncRNAs. (a, b) Volcano plots of DE-lncRNAs of *M* vs. *N* and AS vs. *M*. Blue means downregulated genes, red represents upregulated genes, and black represents genes that do not differ significantly. (c) Heat maps of DE-lncRNAs of 3 groups. Red means high expression, and blue means low expression (*n* = 3).

**Figure 4:** Volcano plots and heat maps of DE-mRNAs. (a, b) Volcano plots of DE-mRNAs of *M* vs. *N* and AS vs. *M*. Blue means downregulated genes, red represents upregulated genes, and black represents genes that do not differ significantly. (c) Heat maps of DE-mRNAs of 3 groups. Red means high expression, and green means low expression (*n* = 3).

**Figure 5:** Coexpression of 237 DE-lncRNAs and 178 DE-mRNAs. Finally, 32 DE-lncRNAs and 13 DE-mRNAs have a targeted regulation relationship. The blue square represents DE-lncRNAs, and the red circle represent their targeted DE-mRNAs.

**Figure 6:** KEGG and GO enrichment analysis of 32 DE-lncRNAs targeted 13 DE-mRNAs. (a) The top 20 pathways in GO enrichment. (b) The top 20 pathways in KEGG enrichment. The red-labeled pathway is the pathway with the highest impact factor (TOP 2 in GO pathway and TOP 1 in KEGG pathway), and the labeled genes are the corresponding DE-mRNAs.

**Figure 7:** The recovery effect of AS on the lncRNAs co-expression profiles. (a–h) qRT-PCR verification of NONRATT028523.2, NONRATT026955.2, NONRATT016111.2, NONRATT028522.2, MSTRG.22291.30, NONRATT022172.2, ENSRNOT00000083625, and MSTRG.15507.1. Columns are mean ± SD (*n* = 3). ^∗^*P* < 0.05, ^∗∗^*P* < 0.01 vs. group *M*.

**Figure 8:** The recovery effect of AS on the mRNAs coexpression profiles. (a–g) qRT-PCR verification of Adipoq, Lpl, Abcd2, Cnr1, Fst, Mapk13, and Zbtb16. Columns are the mean ± SD (*n* = 3). ^∗^*P* < 0.05, ^∗∗^*P* < 0.01 vs. group *M*.

**Table 1:** Primer sequences.

Gene	Forward primer	Reverse primer
NONRATT028522.2	TGTACGTCTCATAAACCCGAAAGCC	GACCGCTGACAAGTCCTCAATGG
NONRATT028523.2	GGAGCCGCTCACATATACTCACTG	CGCCCACCGAGGTTTCTTGATG
NONRATT016111.2	AGAGTGATGTGGGTGTCAGAGACTG	CAGCCGACTAGCTCAAAGGAAACC
NONRATT026955.2	TTGGATTGCCAGCGGTGATAACTC	CTTCAAGTAGGAGTCAGCACGAACC
NONRATT022172.2	AGTTGCCGTGGAATCTTTCAAAAGC	AAGGTTTCCTCTCTAGGCGACTCTG
ENSRNOT00000083625.1	TCGGAGCCAGTAATGAATGTGAACG	CCTGCACGGTCTGCCTTTTATCG
MSTRG.22291.30	ACATTTCAGAGTGGGCAGCAACC	TAACCAGGGCAGGAACCAGACC
MSTRG.15507.1	TGGGTTTCTCGTCTGGTGAATGATG	TCAGTTGGGCTCCTCCTAGTATGTG
Zbtb16	CGCCACCTTCGCTCACATACAG	ACTTCTTGCCACAGCCATTACACTC
Abcd2	AGCGTCCACCTCTACCACATAGTC	TCGTCCAGCAATGCGTACTTCG
Cnr1	GTGTGCTGCTGCTGTTCATTGTG	CGTGTGGATGATGATGCTCTTCTGG
Adipoq	CGCAGGTGTTCTTGGTCCTAAGG	CCCTACGCTGAATGCTGAGTGATAC
Mapk13	TGAAGACACAGCACCTCAGCAATG	GGTGTTCAGCAGGAGGTTGGAAG
LPl	TTCCAAGGAGGCATTTGAGAAAGGG	TGTAGGGCATCTGAGAGCGAGTC
Fst	CTCCGGCGTACTGCTTGAAGTG	GGTCTTCCTCTTCCTCCTCTTCCTC

**Table 2:** Specific information of coexpressed 13 DE-mRNAs and 32 DE-lncRNAs among the three groups.

DE-mRNAs	log2FC		*P* value		Change trend	Coexpressed DE-lncRNAs and change trend (M : N/AS : M)
	M/N	AS/M	M/N	AS/M	(M : N/AS : M)	
Adipoq	-1.068117924	0.662296394	0.001175196	0.014328704	Down/up	MSTRG.27727.3 (down/up); MSTRG.15507.1 (down/up); MSTRG.20388.4 (up/down); MSTRG.22291.30 (up/down); MSTRG.19243.4 (up/down); MSTRG.3358.4 (up/down); MSTRG.17976.2 (up/down); MSTRG.3358.5 (down/up)
Lpl	0.794905651	-0.853559676	1.40585E-05	0.001316594	Up/down	ENSRNOT00000083625 (up/down)
Cnr1	1.356438499	-1.094538823	2.75E-09	0.000440588	Up/down	NONRATT022172.2 (up/down)
Abcd2	-1.158263739	1.597586728	0.049047871	5.70E-05	Down/up	MSTRG.15507.1 (down/up); MSTRG.22291.30 (up/down); MSTRG.6886.9 (up/down); MSTRG.23304.3 (down/up); NONRATT026955.2 (down/up); MSTRG.18510.2 (down/up)
Fst	0.894560311	-1.715392735	0.030006981	0.002178484	Up/down	NONRATT016111.2 (up/down)
Prom2	0.677685369	-0.600170925	5.42E-05	0.000422686	Up/down	NONRATT018580.2 (up/down)
RGD1561730	1.805761687	-1.190334966	0.00210257	0.037622436	Up/down	MSTRG.14467.13 (up/down); MSTRG.6158.10 (up/down); MSTRG.22291.30 (up/down); NONRATT019663.2 (down/up); MSTRG.203.13 (down/up); MSTRG.19772.13 (up/down); MSTRG.23304.3 (down/up); MSTRG.6158.17 (up/down); MSTRG.6158.13 (up/down); MSTRG.21462.2 (up/down); MSTRG.119.2 (down/up); MSTRG.11788.3 (up/down)
Syt13	1.55842082	-1.496316284	3.18E-12	2.80E-05	Up/down	NONRATT018376.2 (up/down)
Mapk13	0.777767762	-0.60268267	0.000106259	0.00169343	Up/down	MSTRG.15507.1 (down/up); MSTRG.22291.30 (up/down); MSTRG.6886.9 (up/down); MSTRG.23304.3 (down/up); NONRATT026955.2 (down/up); MSTRG.18510.2 (down/up)
Zbtb16	2.132334028	-1.354103129	1.17E-15	3.23E-07	Up/down	MSTRG.26690.1 (up/down); NONRATT028523.2 (up/down); NONRATT028522.2 (up/down)
Usp9y	Inf	-6.369845576	5.86E-07	9.01E-06	Up/down	MSTRG.19243.4 (up/down)
Slc4a7	1.327084846	-1.494267287	8.17E-14	6.66E-07	Up/down	NONRATT010755.2 (up/down)
Nek5	1.105543899	-1.069217283	5.11E-07	0.001094649	Up/down	NONRATT011643.2 (up/down)

## Data Availability

The datasets used and analyzed during the current study are available from the corresponding author on reasonable request.

## References

[1] Collins A. J., Foley R. N., Chavers B., Gilbertson D., Agodoa L. (2014). 2013 USRDS annual data report: atlas of chronic kidney disease and end-stage renal disease in the United States. *American Journal of Kidney Diseases*.

[2] Mishra K., Kanduri C. (2019). Understanding long noncoding RNA and chromatin interactions: what we know so far. *Noncoding RNA*.

[3] Leimena C., Qiu H. (2018). Non-coding RNA in the pathogenesis, progression and treatment of hypertension. *International Journal of Molecular Sciences*.

[4] Yao Q. P., Xie Z. W., Wang K. X. (2017). Profiles of long noncoding RNAs in hypertensive rats: long noncoding RNA XR007793 regulates cyclic strain-induced proliferation and migration of vascular smooth muscle cells. *Journal of Hypertension*.

[5] Jin L., Lin X., Yang L. (2018). AK098656, a novel vascular smooth muscle cell-dominant long noncoding RNA, promotes hypertension. *Hypertension*.

[6] Ziaeian B., Fonarow G. C. (2016). Epidemiology and aetiology of heart failure. *Nature Reviews. Cardiology*.

[7] Li C., Lin L., Zhang L. (2021). Long noncoding RNA p21 enhances autophagy to alleviate endothelial progenitor cells damage and promote endothelial repair in hypertension through SESN2/AMPK/TSC2 pathway. *Pharmacological Research*.

[8] Xie H., Xue J. D., Chao F., Jin Y. F., Fu Q. (2016). Long non-coding RNA-H19 antagonism protects against renal fibrosis. *Oncotarget*.

[9] Tian H., Wu M., Zhou P., Huang C., Ye C., Wang L. (2018). The long non-coding RNA MALAT1 is increased in renal ischemia-reperfusion injury and inhibits hypoxia-induced inflammation. *Renal Failure*.

[10] Xiang Y., Zhang Y., Tang Y., Li Q. (2017). MALAT1 modulates TGF-*β*1-induced endothelial-to-mesenchymal transition through downregulation of miR-145. *Cellular Physiology and Biochemistry*.

[11] Shahzad M., Shabbir A., Wojcikowski K., Wohlmuth H., Gobe G. C. (2016). The antioxidant effects of radix Astragali (Astragalus membranaceus and related species) in protecting tissues from injury and disease. *Current Drug Targets*.

[12] Che X., Wang Q., Xie Y. (2015). Astragaloside IV suppresses transforming growth factor-*β*1 induced fibrosis of cultured mouse renal fibroblasts via inhibition of the MAPK and NF-*κ*B signaling pathways. *Biochemical and Biophysical Research Communications*.

[13] Li W., Sun W., Yang C. H., Hu H. Z., Jiang Y. H. (2014). Tanshinone II a protects against lipopolysaccharides-induced endothelial cell injury via Rho/Rho kinase pathway. *Chinese Journal of Integrative Medicine*.

[14] Han C., Jiang Y. H., Li W., Liu Y., Qi Z. Q. (2019). Study on the antihypertensive mechanism of Astragalus membranaceus and salvia miltiorrhiza based on intestinal Flora-host metabolism. *Evidence-based Complementary and Alternative Medicine*.

[15] Li W., Jiang Y. H., Wang Y. (2020). Protective effects of combination of radix astragali and radix salviae miltiorrhizae on kidney of spontaneously hypertensive rats and renal intrinsic cells. *Chinese Journal of Integrative Medicine*.

[16] Hou G., Jiang Y., Zheng Y. (2021). Mechanism of radix astragali and radix salviae miltiorrhizae ameliorates hypertensive renal damage. *BioMed Research International*.

[17] Han C., Jiang Y. H., Li W., Liu Y. (2021). Astragalus membranaceus and salvia miltiorrhiza ameliorates cyclosporin A-induced chronic nephrotoxicity through the "gut-kidney axis". *Journal of Ethnopharmacology*.

[18] Liu Y., Jiang Y., Li W., Han C., Qi Z. (2020). MicroRNA and mRNA analysis of angiotensin II-induced renal artery endothelial cell dysfunction. *Experimental and Therapeutic Medicine*.

[19] Fang S., Sigmund C. D. (2020). PPAR*γ* and RhoBTB1 in hypertension. *Current Opinion in Nephrology and Hypertension*.

[20] Gu D., Fang D., Zhang M. (2021). Gastrin, via activation of PPAR*α*, protects the kidney against hypertensive injury. *Clinical Science (London, England)*.

[21] Kirkby N. S., Sampaio W., Etelvino G. (2018). Cyclooxygenase-2 selectively controls renal blood flow through a novel PPAR*β*/*δ*-dependent vasodilator pathway. *Hypertension*.

[22] Miyamoto S., Sharma K. (2013). Adipokines protecting CKD. *Nephrology, Dialysis, Transplantation*.

[23] Tian M., Tang L., Wu Y., Beddhu S., Huang Y. (2018). Adiponectin attenuates kidney injury and fibrosis in deoxycorticosterone acetate-salt and angiotensin II-induced CKD mice. *American Journal of Physiology. Renal Physiology*.

[24] Wu F., Huang J., Zhou J. (2019). Inverse correlation between serum adiponectin level and albuminuria in pregnancy-induced hypertension patients. *Clinical and Experimental Hypertension*.

[25] Wu S. A., Kersten S., Qi L. (2021). Lipoprotein lipase and its regulators: an unfolding story. *Trends in Endocrinology and Metabolism*.

[26] Olivecrona G. (2016). Role of lipoprotein lipase in lipid metabolism. *Current Opinion in Lipidology*.

[27] Dao M., François H. (2021). Cannabinoid receptor 1 inhibition in chronic kidney disease: a new therapeutic toolbox. *Frontiers in Endocrinology*.

[28] Chung K. W., Lee E. K., Lee M. K., Oh G. T., Yu B. P., Chung H. Y. (2018). Impairment of PPAR*α*and the fatty acid oxidation pathway aggravates renal fibrosis during aging. *Journal of the American Society of Nephrology*.

[29] Kang H. M., Ahn S. H., Choi P. (2015). Defective fatty acid oxidation in renal tubular epithelial cells has a key role in kidney fibrosis development. *Nature Medicine*.

[30] Wei S., Zhang M., Zheng Y., Yan P. (2018). ZBTB16 overexpression enhances white adipogenesis and induces brown-like adipocyte formation of bovine white intramuscular preadipocytes. *Cellular Physiology and Biochemistry*.

[31] Cheng Z., Tu J., Zhang H., Zhou B. (2021). Urolithin A attenuates renal fibrosis by inhibiting TGF-*β*1/Smad and MAPK signaling pathways. *Journal of Functional Foods*.

[32] Morita M., Shimozawa N., Kashiwayama Y., Suzuki Y., Imanaka T. (2011). ABC subfamily D proteins and very long chain fatty acid metabolism as novel targets in adrenoleukodystrophy. *Current Drug Targets*.

